The article "Suppression of epileptogenesis-associated changes in response to seizures in FGF22-deficient mice" was retracted in 2023. Reasons: duplicated images; unreliable results or conclusions; concerns about the data.

# Suppression of epileptogenesis-associated changes in response to seizures in FGF22-deficient mice

**DOI:** 10.3389/fncel.2013.00043

**Published:** 2013-04-18

**Authors:** Clara H. Lee, Hisashi Umemori

**Affiliations:** ^1^Molecular and Behavioral Neuroscience Institute, University of Michigan Medical School Ann Arbor, MI, USA; ^2^Department of Biological Chemistry, University of Michigan Medical School Ann Arbor, MI, USA

**Keywords:** fibroblast growth factor 22, temporal lobe epilepsy, neurogenesis, hilar ectopic dentate granule cells, hilar cell death, mossy fiber sprouting

## Abstract

In the developing hippocampus, fibroblast growth factor (FGF) 22 promotes the formation of excitatory presynaptic terminals. Remarkably, FGF22 knockout (KO) mice show resistance to generalized seizures in adults as assessed by chemical kindling, a model that is widely used to study epileptogenesis (Terauchi et al., 2010). Repeated injections of low dose pentylenetetrazol (PTZ) induce generalized seizures (“kindled”) in wild type (WT) mice. With additional PTZ injections, FGF22KO mice do show moderate seizures, but they do not kindle. Thus, analyses of how FGF22 impacts seizure susceptibility will contribute to the better understanding of the molecular and cellular mechanisms of epileptogenesis. To decipher the roles of FGF22 in the seizure phenotype, we examine four pathophysiological changes in the hippocampus associated with epileptogenesis: enhancement of dentate neurogenesis, hilar ectopic dentate granule cells (DGCs), increase in hilar cell death, and formation of mossy fiber sprouting (MFS). Dentate neurogenesis is enhanced, hilar ectopic DGCs appeared, and hilar cell death is increased in PTZ-kindled WT mice relative to PBS-injected WT mice. Even in WT mice with fewer PTZ injections, which showed only mild seizures (so were not kindled), neurogenesis, hilar ectopic DGCs, and hilar cell death are increased, suggesting that mild seizures are enough to induce these changes in WT mice. In contrast, PTZ-injected FGF22KO mice do not show these changes despite having moderate seizures: neurogenesis is rather suppressed, hilar ectopic DGCs do not appear, and hilar cell death is unchanged in PTZ-injected FGF22KO mice relative to PBS-injected FGF22KO mice. These results indicate that FGF22 plays important roles in controlling neurogenesis, ectopic migration of DGCs, and hilar cell death after seizures, which may contribute to the generalized seizure-resistant phenotype of FGF22KO mice and suggests a possibility that inhibition of FGF22 may alleviate epileptogenesis.

## Introduction

Epilepsy is one of the most common neurological disorders, which is characterized by recurrent seizures. Currently, the only available pharmacological treatments for epilepsy are seizure suppressants. These anticonvulsants may control seizures with various success rates among the different forms of epilepsy. Temporal lobe epilepsy (TLE), which is the most common type of epilepsy in adults, is one of the most refractory epilepsies—about one-third of patients are resistant to pharmacological treatments (Semah et al., 1998; Brodie, 2005; French, 2007). Not only are seizure suppressants often ineffective against intractable epilepsy, they only address the symptoms of the disease and neither prevent its initial development nor stop its progression (McNamara, 1994; Brodie, 2005; French, 2007). In order to develop effective treatment of epilepsy, further understanding of the epileptogenic mechanisms is required.

The article "Suppression of epileptogenesis-associated changes in response to seizures in FGF22-deficient mice" was retracted in 2023. Reasons: duplicated images; unreliable results or conclusions; concerns about the data.

The hippocampus is one of the epileptogenic regions (foci) in TLE and has been a target region for studies on cellular mechanisms of epileptogenesis (McNamara, 1994; Morimoto et al., 2004). Brain insults such as trauma, seizure, stroke, and infection may cause various changes in the hippocampus, which may eventually result in TLE (Pitkänen and Lukasiuk, 2011). Many possible mechanisms have been proposed that might be involved in the process of epileptogenesis (Simonato et al., 2006; Pitkänen and Lukasiuk, 2011), including four changes in the hippocampus that have been widely accepted to be associated with epileptogenesis (Dudek and Sutula, 2007; Parent, 2007): (1) increased neurogenesis in the dentate gyrus (DG), (2) hilar ectopic dentate granule cells (DGCs), (3) loss of hilar cells (interneurons and mossy cells), and (4) formation of mossy fiber sprouting (MFS). These changes are proposed to be induced by brain insults, which may result in the rewiring of the hippocampal network to establish a possible epileptic circuitry (McNamara, 1994; Coulter, 2001; Morimoto et al., 2004; Rakhade and Jensen, 2009; Kokaia, 2011). Increased neurogenesis and hilar ectopic DGCs may contribute to abnormal incorporation of DGCs into the circuitry (Parent et al., 2006; Jessberger et al., 2007; Walter et al., 2007; Kron et al., 2010), loss of hilar cells may disrupt existing physiological balance in the network (Dudek and Sutula, 2007; Jiao and Nadler, 2007), and MFS, where sprouted mossy fibers form synapses onto DGCs themselves, may induce recurrent excitation of the DGCs (Sutula et al., 1989; Koyama and Ikegaya, 2004; Morimoto et al., 2004). All of the four mechanisms could cause hyperexcitation of the brain by rearranging the circuitry of the hippocampus. Therefore, understanding of the molecular mechanisms that are responsible for these epileptogenesis-associated events may help identify possible drug targets for the treatment of epilepsy.

The article "Suppression of epileptogenesis-associated changes in response to seizures in FGF22-deficient mice" was retracted in 2023. Reasons: duplicated images; unreliable results or conclusions; concerns about the data.

Growth factors such as neurotrophins and fibroblast growth factors (FGFs) are suggested to be involved in epileptogenesis (Simonato et al., 2006). For example, overexpression of FGF2 increases seizure susceptibility and reduces seizure-induced cell death (Zucchini et al., 2008). Application of BDNF and FGF2 reduces MFS and spontaneous seizures (Paradiso et al., 2009, 2011). MFS arises in the absence of FGF7 (Lee et al., 2012). Thus, growth factors may be crucial molecules to regulate epileptogenesis. We have recently identified a member of FGFs, FGF22 as a molecule that organizes excitatory presynaptic differentiation in the hippocampus (Umemori et al., 2004; Terauchi et al., 2010). Remarkably, we found that FGF22 knockout (KO) mice are resistant to generalized seizures induced by chemical kindling with repeated injections of low dose pentylenetetrazol (PTZ), a GABA receptor antagonist. We therefore asked whether the four epileptogenesis-associated changes—increased DG neurogenesis, hilar ectopic DGCs, hilar cell loss, and MFS—are induced in the hippocampus of FGF22KO mice in response to PTZ injections, in order to get insight into the cellular basis of their seizure-resistant phenotype. We here show that in FGF22KO mice, these changes do not occur, even with moderate seizures after prolonged PTZ injections. Our results suggest that inactivation of FGF22 may increase resistance to epileptogenesis-associated changes in response to seizures in the hippocampus and that FGF22 could be a potential target for treatment of epilepsy.

## Materials and methods

### Animals

FGF22KO mice were described previously (Terauchi et al., 2010). FGF22KO mice have been backcrossed with C57BL/6 for more than 15 generations. Five-month-old FGF22KO mice and C57BL/6 mice [wild type (WT)] were used in this study. Genotypes of the mice were verified by genomic PCR. Male mice were used. The numbers of animals used in this study are shown in Figure 1B. All animal use and care was in accordance with the institutional guidelines and was approved by the University Committee on Use and Care of Animals.

**Figure 1:** **Characteristics of the three animal groups used in this study: non-kindled WT mice with mild seizures, kindled WT mice, and non-kindled FGF22KO mice with moderate seizures.** WT and FGF22KO mice were injected with a GABA receptor antagonist pentylenetetrazol (PTZ; 35 mg/kg) every 48 h to induce seizures. Control animals received PBS. **(A)** Typical time course of seizure development and three animal groups. Group 1: WT mice were injected until they first showed a seizure greater then level 1 (~14 PTZ injections); Group 2: WT mice were injected until they were kindled (~24 PTZ injections); Group 3: FGF22KO mice were injected with PTZ for 37 times—they showed moderate seizures but did not kindle. **(B)** Summary of characteristics of three animal groups. For each mouse group, the genotype, the highest seizure level, kindled or not, the cumulative seizure score, and the number of animals are shown. The highest seizure level indicates the most severe seizure level observed over the entire injection period. Group 1 mice showed only mild seizures (one level 3 seizure), Group 2 mice showed severe seizures (level 6 = kindled), and Group 3 mice showed mild to moderate seizures (level 3–4). The cumulative seizure score is the sum of seizure levels that the mouse has experienced throughout the injection period. Group 1 mice received considerably less cumulative seizures relative to Groups 2 and 3, which received comparable amount of cumulative seizures to each other.

The article "Suppression of epileptogenesis-associated changes in response to seizures in FGF22-deficient mice" was retracted in 2023. Reasons: duplicated images; unreliable results or conclusions; concerns about the data.

### Kindling and animal groups

PTZ (35 mg/kg), a GABA receptor antagonist, was injected intraperitoneally every 48 h in WT and FGF22KO mice to induce seizures. Control animals received PBS. The mice were observed for an hour after each PTZ injection, and the maximum level of seizure within the hour was recorded. The seizure responses were noted on a revised Racine's scale for PTZ kindling (Lüttjohann et al., 2009) as follows: Stage 0: No seizure observed; Stage 1: Sudden behavioral arrest and/or motionless staring; Stage 2: Facial jerking with muzzle or muzzle and eye; Stage 3: Neck jerks; Stage 4: Clonic seizure in a sitting position; Stage 5: Convulsions including clonic and/or tonic–clonic seizures while lying on the belly and/or pure tonic seizures; Stage 6: Convulsions including clonic and/or tonic–clonic seizures while lying on the side and/or wild jumping. Mice were defined as “kindled” when they displayed either one class 6 seizure or two successive class 5 seizures. We prepared three animal groups (the number of mice in each group is shown in Figure 1B) that are different in genotype and seizure levels for the study (see Figure 1). Group 1: WT mice with mild seizures—WT mice were injected until they first showed a seizure greater then level 1 (average PTZ injections = 14); Group 2: WT mice with kindled seizures—WT mice were injected until they were kindled (average PTZ injections = 24); Group 3: FGF22KO mice with moderate seizures (not kindled)—FGF22KO mice were injected with PTZ 37 times; the mice showed moderate seizures but did not kindle.

### Brain sectioning

The mice were perfused with 4% paraformaldehyde (PFA). The brains were dissected and post-fixed in 4% PFA for 24 h. The brains were then placed in 30% sucrose solution for 48 h, frozen, and stored at −80°C. The sections from the same region of the hippocampus were used (4–6 sections/mouse) in this study in order to standardize quantification of the cell numbers. Sections between 2.5 and 3.5 mm from the midline were used for the study. Each section was 20 μm thick.

The article "Suppression of epileptogenesis-associated changes in response to seizures in FGF22-deficient mice" was retracted in 2023. Reasons: duplicated images; unreliable results or conclusions; concerns about the data.

### Immunohistochemistry

The sections were blocked in 2% BSA, 2% normal goat serum, and 0.1% TritonX-100 for 30 min, followed by the incubation with primary antibodies for 2 h at room temperature. Secondary antibodies were then applied for 1 h at room temperature, and slides were mounted with p-phenylenediamine. Antibodies used were: DCX (Abcam, ab18723; dilution 1:500), Ki67 (Abcam, ab15580; dilution 1:200), Prox1 (Millipore, MAB5256; dilution 1:250), NeuN (Millipore, MAB377; dilution 1:1000), and ZnT3 (Synaptic Systems, #197002, dilution 1:200). DAPI was added to each section as a nuclear stain. The stained sections were observed under the Olympus BX61 fluorescent microscope. The images were taken with the F-View Soft Imaging System camera.

### Neurogenesis

Neurogenesis within the DGC layer was assessed using immunohistochemistry for doublecortin (DCX), a marker for immature neurons, and Ki67, a marker for proliferating cells. DCX and Ki67 positive cells were counted from the entire DGC layer on a section and divided by the total number of DGCs stained with DAPI.

### Hilar ectopic DGCs

Ectopic DGCs in the hilus were assessed using immunohistochemistry for Prox1, a marker for DGCs. Ectopic location was defined as greater than or equal to two cell body widths outside the granule cell layer (Kron et al., 2010). The number of ectopic Prox1-positive cells was quantified from the entire hilar region of a hippocampal section.

### Hilar cell death

Cell death in the hilus was evaluated by quantifying the number of surviving neurons with immunohistochemistry for NeuN, a marker for mature neurons. The number of NeuN-positive cells was quantified from the entire hilar region of a hippocampal section. The number of hilar ectopic DGCs was subtracted from the number of NeuN-positive cells to evaluate hilar cell death.

### Mossy fiber sprouting

MFS was examined by staining hippocampal sections for ZnT3, a zinc transporter enriched in mossy fibers. The presence of MFS in the inner molecular layer of the DG was examined.

## Results

### FGF22KO mice show moderate seizures but do not kindle with prolonged injections of PTZ

We have previously found that FGF22KO mice are resistant to generalized seizures induced by PTZ kindling (Terauchi et al., 2010), in which we injected animals with PTZ every 48 h to induce generalized (kindled) seizures. In that experiment, when about half of WT mice were kindled (level 6 seizure; after about 21 PTZ injections), no FGF22KO mice were kindled. Here, we first tested if prolonged PTZ injections can make FGF22KO mice kindled. With additional PTZ injections, FGF22KO mice did show mild to moderate (levels 1–4) seizures (Figure 1A). However, even after 37 PTZ injections, they did not kindle. We stopped after 37 PTZ injections, because the cumulative seizure score (the sum of all the seizure levels that the mouse has experienced) for the FGF22KO mouse became ~55 (Figure 1B), which was similar to the one for the kindled WT mouse (~53) (see below).

The article "Suppression of epileptogenesis-associated changes in response to seizures in FGF22-deficient mice" was retracted in 2023. Reasons: duplicated images; unreliable results or conclusions; concerns about the data.

### Preparation of three animal groups to understand the role of FGF22 in epileptogenesis

Since FGF22KO mice do not kindle even with prolonged PTZ injections, we designed experiments to address the cellular basis of their kindled seizure-resistant phenotype. We focused on four epileptogenesis-associated changes: enhanced DG neurogenesis, hilar ectopic DGCs, hilar cell loss, and MFS. For our experiments, it was important to consider the possibility that the levels of these changes may correlate with the amount of seizure overtime that the animal experienced in response to PTZ injections. Because FGF22KO mice do not kindle, direct comparison between kindled WT mice and non-kindled FGF22KO mice may not be conclusive. Therefore, to understand the role of FGF22 in the epileptogenesis-associated changes apart from the effects of seizure activities on them, we injected FGF22KO mice with PTZ until their cumulative seizure score becomes equivalent to that of kindled WT mice so that FGF22KO mice experience similar overall amount of seizure activity to kindled WT mice. Yet, these two groups of animals still differ in the highest seizure level experienced (level 3–4 moderate seizures for FGF22KO mice as opposed to level 6 kindled seizures for WT mice). Thus, we prepared another group of WT mice with only mild, non-kindled seizures. Together, we prepared three groups of animals for our experiments (Figure 1B)—Group 1, WT mice with mild seizures (not kindled with just one level 3 seizure; cumulative seizure score = 8.4); Group 2, kindled WT mice (with level 6 seizures; cumulative seizure score = 52.5); and Group 3, FGF22KO mice with moderate seizures (not kindled with up to level 4 seizures; cumulative seizure score = 55.4). By comparing epileptogenesis-associated changes happening in these three groups, we can evaluate the contribution of both the genotype and the seizures that animals experienced. For each group, we also prepared a control group of mice, which received PBS instead of PTZ for the same durations.

The article "Suppression of epileptogenesis-associated changes in response to seizures in FGF22-deficient mice" was retracted in 2023. Reasons: duplicated images; unreliable results or conclusions; concerns about the data.

### Dentate neurogenesis increases in WT mice with mild or kindled seizures, but decreases in FGF22KO mice with moderate seizures

Enhanced neurogenesis in the DG is implicated in epileptogenesis because it may lead to aberrant integration of DGCs (Parent et al., 2006; Jessberger et al., 2007; Walter et al., 2007; Kron et al., 2010). We first assessed the level of cell proliferation in the DGC layer by staining hippocampal sections prepared from the three groups of mice with Ki67, a marker of proliferating cells (Figure 2). The sections from the same region of the hippocampus were used in order to standardize quantifications of cell numbers. At the basal level (PBS-injected mice), there was no significant difference in the number of Ki67-positive cells in the DG between WT and FGF22KO mice (Figure 2B). The number of Ki67-positive cells was increased in kindled WT mice relative to PBS-injected controls. It was increased more dramatically in non-kindled WT mice with mild seizures, suggesting that mild seizures enhance cell proliferation in the DG in WT mice. In contrast, FGF22KO mice showed a decrease in the number of Ki67-positive cells in the DG when injected with PTZ, despite having moderate seizures (Figure 2).

**Figure 2:** **The number of proliferating cells in the DG increases in WT mice but decreases in FGF22KO mice upon PTZ injections.** Region-matched sagittal hippocampal sections were prepared from PBS- and PTZ-injected WT and FGF22KO mice (3 groups of mice as shown in Figure 1) and stained for Ki67, a marker for proliferating cells. **(A)** Ki67 positive cells (pink) with DAPI (blue) in the DG of PBS- or PTZ-injected WT and FGF22KO mice. **(B)** Quantification of the numbers of Ki67-positive cells in the DGC layer per section in PBS-injected WT and FGF22KO mice (n.s. = not significant). **(C)** Quantification of the percentages of Ki67-positive cells in DGCs. Data are normalized against corresponding PBS controls. The percentage of Ki67-positive cells was significantly increased in WT mice with mild and kindled seizures, but was decreased in FGF22KO mice with moderate seizures upon PTZ-injections. Bars are mean ± s.e.m. Data are from 4–6 sections from 3–10 mice (see Figure 1B) per each condition. Student's *t*-test *P*-values are indicated.

Similar but slightly different results were observed with staining for DCX, a marker of immature neurons (Figure 3). At the basal level (PBS-injected mice), we found less DCX-positive cells in the DG in FGF22KO mice than in WT mice (Figure 3B), suggesting that FGF22 is involved in neuronal differentiation. The number of DCX-positive cells was increased in WT mice with kindled seizures, which is consistent with previous reports (Parent et al., 2006; Jessberger et al., 2007; Yin et al., 2007; Buga et al., 2012). It was similarly increased in WT mice with mild seizures. These, together with the Ki67 results suggest that seizures induce neurogenesis, but mild seizures affect more on proliferation than kindled seizures do. In contrast, the number of DCX-positive cells was decreased in FGF22KO mice with moderate seizures. These results suggest that FGF22 is involved in seizure-induced increases in neurogenesis in the DG.

The article "Suppression of epileptogenesis-associated changes in response to seizures in FGF22-deficient mice" was retracted in 2023. Reasons: duplicated images; unreliable results or conclusions; concerns about the data.

**Figure 3:** **The number of immature neurons in the DG is increased in WT mice with mild and kindled seizures, but is decreased in FGF22KO mice with moderate seizures.** Region-matched sagittal hippocampal sections were prepared from PBS- and PTZ-injected WT and FGF22KO mice (3 groups of mice as shown in Figure 1) and stained for doublecortin (DCX), a marker for immature neurons. **(A)** DCX positive cells (green) with DAPI (blue) in the DG of PBS- or PTZ-injected mice. **(B)** Quantification of the numbers of DCX-positive cells in the DGC layer per section in PBS-injected WT and FGF22KO mice. **(C)** Quantification of the percentages of DCX-positive cells in DGCs. Data are normalized against corresponding PBS controls. Neurogenesis, as reflected by the percentage of DCX-positive cells, was significantly increased in WT mice with mild and kindled seizures, but was decreased in FGF22KO mice with moderate seizures upon PTZ-injections. Bars are mean ± s.e.m. Student's *t*-test *P*-values are indicated.

### Hilar ectopic DGCs appear in WT mice with mild or kindled seizures, but not in FGF22KO mice with moderate seizures

Hilar ectopic DGCs may lead to aberrant integration of DGCs and contribute to epileptogenesis (Parent et al., 2006; Jessberger et al., 2007; Walter et al., 2007; Kron et al., 2010). We next examined the number of hilar ectopic DGCs by staining hippocampal sections for Prox1, a marker of DGCs (Figure 4). There was no hilar ectopic DGC in the basal condition (PBS injected) in both WT and FGF22KO mice. The number of hilar ectopic DGCs dramatically increased in WT mice with kindled seizures (Figure 4B). It was also substantially increased in WT mice with mild seizures. However, there was no significant increase in FGF22KO mice with moderate seizures. These results suggest that FGF22 is involved in ectopic migration of DGCs in response to seizures.

**Figure 4:** **The number of hilar ectopic DGCs is increased in WT mice with mild and kindled seizures, but not in FGF22KO mice with moderate seizures.** Region-matched sagittal hippocampal sections were prepared from PBS- and PTZ-injected WT and FGF22KO mice (3 groups of mice as shown in Figure 1) and stained for Prox1, a marker for DGCs. Ectopic location was defined as greater than or equal to two cell body widths outside the granule cell layer. **(A)** Prox1 positive cells in the DG and hilus of PBS- or PTZ-injected mice. **(B)** Quantification of the numbers of ectopic Prox1-positive cells in the hilus. The number of hilar ectopic DGCs was significantly increased in WT mice with mild and kindled seizures, but not in FGF22KO mice with moderate seizures upon PTZ-injections. Bars are mean ± s.e.m. Student's *t*-test *P*-values are indicated.

The article "Suppression of epileptogenesis-associated changes in response to seizures in FGF22-deficient mice" was retracted in 2023. Reasons: duplicated images; unreliable results or conclusions; concerns about the data.

### Hilar cell death increases in WT mice with mild or kindled seizures, but is unchanged in FGF22KO mice with moderate seizures

An increase in hilar cell death is another change that is associated with epileptogenesis (Dudek and Sutula, 2007; Jiao and Nadler, 2007). We next evaluated the level of hilar cell death in PTZ-injected WT and FGF22KO mice by quantifying the number of surviving mature neurons in the hilar region with NeuN staining (Figure 5). We have calculated the number of hilar cells by subtracting the number of hilar ectopic DGCs (Figure 4) from the number of NeuN-positive cells. The number of hilar cells was decreased in kindled WT mice relative to PBS-injected mice, which is consistent with previous reports (Sloviter, 1983; Dudek and Sutula, 2007; Jiao and Nadler, 2007; Naseer et al., 2013). It was also decreased in non-kindled WT mice with mild seizures, suggesting that similar to the case of neurogenesis (Figures 2, 3), mild seizures are enough to increase hilar cell death in WT mice. However, the number of hilar cells was not significantly changed in PTZ-injected FGF22KO mice with moderate seizures relative to PBS-injected controls. These results suggest that FGF22 plays important roles in increasing hilar cell death in response to seizures.

**Figure 5:** **Hilar cell death is increased in WT mice with mild and kindled seizures, but is unchanged in FGF22KO mice with moderate seizures.** Region-matched sagittal hippocampal sections were prepared from PBS- and PTZ-injected WT and FGF22KO mice (3 groups of mice as shown in Figure 1) and stained for NeuN, a marker for mature neurons. **(A)** NeuN staining of the hilar sections from PBS- or PTZ-injected mice. **(B)** Quantification of the numbers of NeuN-positive cells in the hilus per section in PBS-injected WT and FGF22KO mice. **(C)** Quantification of the numbers of hilar cells. To evaluate hilar cell number, the number of hilar ectopic DGCs (Figure 4) was subtracted from the number of NeuN-positive cells. Data are normalized relative to the corresponding PBS control. After PTZ injections, the number of hilar cells significantly decreased in WT mice both with mild and with kindled seizures, but not in FGF22KO mice with moderate seizures. Bars are mean ± s.e.m. *P*-values by Student's *t*-test are indicated.

The article "Suppression of epileptogenesis-associated changes in response to seizures in FGF22-deficient mice" was retracted in 2023. Reasons: duplicated images; unreliable results or conclusions; concerns about the data.

### MFS is induced only in kindled WT mice

In TLE patients and animal models of TLE, mossy fibers (axons of DGCs) often abnormally sprout to the dentate molecular layer and form excitatory synapses with the dendrites of DGCs (MFS). Accordingly, MFS may induce recurrent excitation of DGCs and contribute to epileptogenesis. We next examined whether WT and FGF22KO mice display MFS after seizures. To examine MFS, we stained DG sections with ZnT3, a zinc transporter that is abundant in mossy fiber terminals (Wenzel et al., 1997). MFS in the dentate molecular layer was detected in kindled WT mice (Figure 6), as observed previously with Timm staining (Sutula et al., 1989; Cavazos et al., 1991; Parent et al., 1999). In contrast, MFS was not detected in non-kindled WT mice with mild seizures, suggesting that more severe or prolonged seizures may be required to form MFS in WT mice. MFS was not observed in FGF22KO mice with moderate seizures either. This implies that either FGF22 is required for the formation of MFS or that more severe seizures are necessary to induce MFS.

**Figure 6:** **MFS is only induced in kindled WT mice.** Region-matched sagittal hippocampal sections were prepared from PBS- and PTZ-injected WT and FGF22KO mice (3 groups of mice as shown in Figure 1) and stained for ZnT3, a zinc transporter enriched in mossy fiber terminals, to examine MFS in the DG. Kindled WT mice show MFS in the dentate molecular layer (arrows), while non-kindled WT and FGF22KO mice do not.

## Discussion

FGF22KO mice are more resistant to generalized seizures than WT mice as assessed by PTZ kindling (Terauchi et al., 2010). Here we addressed the possible cellular basis for the phenotype by focusing on four changes in the hippocampus associated with epileptogenesis: enhancement of dentate neurogenesis, appearance of hilar ectopic DGCs, increase in hilar cell death, and formation of MFS. These changes were indeed observed in kindled WT mice. Even in non-kindled WT mice with only mild seizures, three changes, enhanced neurogenesis, hilar ectopic DGCs, and increased hilar cell death, occurred. In contrast, PTZ-injected FGF22KO mice did not show any of these four changes, despite having moderate seizures after prolonged injections of PTZ. From these results, we conclude that FGF22 plays critical roles in increasing neurogenesis, ectopic DGCs, and hilar cell death in response to seizures. As for MFS, since MFS was not detected in WT mice with mild seizures either, we conclude that either FGF22 is involved in the formation of MFS or that more severe seizures are necessary to induce MFS. Our results suggest that inhibition of FGF22 suppresses neurogenesis, hilar ectopic DGCs, and hilar cell death (and possibly MFS) in response to seizures.

The article "Suppression of epileptogenesis-associated changes in response to seizures in FGF22-deficient mice" was retracted in 2023. Reasons: duplicated images; unreliable results or conclusions; concerns about the data.

Since FGF22KO mice did show moderate seizures in our experiments, suppression of epileptogenesis-associated changes in FGF22KO mice is not due to lack of seizures, but rather due to FGF22-deficiency. Thus, our results indicate that FGF22 is involved in seizure activity-induced modifications in the hippocampus. We have previously shown that FGF22 from CA3 pyramidal neurons promotes the organization of excitatory synapses formed onto them (Terauchi et al., 2010). FGF22 from CA3 may also send signals to DGCs to regulate neurogenesis and hilar cell survival in an activity-dependent manner. FGF22-dependent signals may induce other growth factors, neurotrophins, morphogens, and cytokines that are implicated in dentate neurogenesis and cell survival (Simonato et al., 2006; Parent, 2007; Zhao et al., 2008). We are currently indentifying FGF22 receptors and downstream signals mediating these epileptogenesis-associated changes using FGF receptor mutants and are analyzing the roles of FGF22-target genes in dentate neurogenesis.

Another interesting finding is that in FGF22KO mice with moderate seizures, neurogenesis is decreased, rather than unchanged as was seen in the case of hilar cell death. One possible interpretation for this finding is that seizure activities might eventually be generating two signals, positive signals resulting in reactive neurogenesis and negative signals for negative-feedback/homeostatic-control, to regulate dentate neurogenesis and that FGF22 is preferentially involved in the positive signals. Further analysis should reveal the activity-dependent signaling pathways that regulate neurogenesis.

Most importantly, our results suggest a possibility that FGF22 inactivation could suppress the enhancement of neurogenesis, ectopic DGCs, and hilar cell death (and possibly MFS) in response to seizures. Thus, FGF22 may join FGF2 as the FGFs that are involved in epileptogenesis or epileptogenesis-associated changes. It has been shown that aberrant adult-born DGCs can cause epilepsy (Pun et al., 2012), hilar cell death causes DGC hyperexcitability (Jinde et al., 2012), and MFS is likely to contribute to seizure susceptibility (Morgan et al., 2007). Thus, targeting FGF22 could offer a novel strategy to prevent epileptogenesis or epileptogenesis-associated changes. For this reason, we are currently performing small molecule screening for FGF22 inhibitors, hoping to identify candidate drugs to treat or alleviate TLE.

The article "Suppression of epileptogenesis-associated changes in response to seizures in FGF22-deficient mice" was retracted in 2023. Reasons: duplicated images; unreliable results or conclusions; concerns about the data.

### Conflict of interest statement

The authors declare that the research was conducted in the absence of any commercial or financial relationships that could be construed as a potential conflict of interest.
